RETRACTED

# Clinical and Biological Significances of a Ferroptosis-Related Gene Signature in Lung Cancer Based on Deep Learning

**DOI:** 10.1155/2022/6495301

**Published:** 2022-08-25

**Authors:** Xiaosong Yang, Xuanjian Hu, Na Guo

**Affiliations:** ^1^Department of Anesthesiology, Sun Yat-sen University Cancer Center, State Key Laboratory of Oncology in South China, Collaborative Innovation Center for Cancer Medicine, 651 Dongfengdong Road, Guangzhou 510060, China; ^2^Guangdong Esophageal Cancer Institute, Guangzhou 510060, China

## Abstract

Acyl-CoA synthetase long-chain family member 4 (ACSL4) has been linked to the occurrence of tumors and is implicated in the ferroptosis process. Deep learning has been applied to many areas in health care, including imaging diagnosis, digital pathology, classification of cancer, and prediction of metastasis. Nonetheless, neither the level of ACSL4 expression nor its predictive significance in non-small-cell lung cancer (NSCLC) is well understood at this time. Predictions of the ACSL4 mRNA expressions in NSCLC and its link to NSCLC prognosis were made with the aid of the Oncomine and TCGA databases. By performing real-time PCR, we detected the levels of ACSL4 expression that were present in human NSCLC samples. Analyses of the diagnostic, as well as the prognostic significance of ACSL4 in NSCLC, were performed with the use of Kaplan-Meier curves. To assess the influence of ACSL4 on ferroptosis in NSCLC cell lines, an inducer of ferroptosis, namely, erastin, was utilized in this study. In NSCLC tissues, there was a substantial decrease in the level of ACSL4 expression (*p* < 0.001), and this was in line with the findings of the inquiry into the Oncomine and TCGA databases. After that, the findings of the immunohistochemistry analysis revealed that the ACSL4 staining was weakened in NSCLC samples in contrast with the normal samples. It was shown that the differential expression of ACSL4 was substantially linked to the stages of cancer, smoking behaviors, and the status of nodal metastases (all *p* < 0.001). According to the findings of the survival analysis, both RFS and OS were favorable among NSCLC patients who had elevated expression of ACSL4. The ferroptosis sensitization in cancer cells may be reestablished with upregulation of ACSL4 through gene transfection. Mechanistically, protein ubiquitination could perform a remarkable function in ACSL4-induced ferroptosis. ACSL4, which has a function in ferroptosis as both a contributor and monitor, was shown to be downregulated in NSCLC. This finding suggests that ACSL4 might function as a helpful diagnostic and prognostic biological marker and might also be considered a novel possible treatment target for NSCLC.

RETRACTED

## 1. Introduction

Lung cancer is the most prevalent type of malignancy worldwide and the major contributor to cancer-associated fatalities [1]. Lung cancer is divided into small-cell lung cancer (SCLC) and non-small-cell lung cancer (NSCLC). In the case of NSCLC, it is further classified into squamous cell carcinoma (SCC) and adenocarcinoma (ADC) which is responsible for the highest percentage of all lung cancer cases [2]. The processes that drive the growth of tumors in NSCLC and the treatment approaches that might be implemented are still important research topics.

Cancer cells often exhibit innate or acquired resistance to the programmed cell death process known as apoptosis. As a result, the identification of nonapoptotic types of regulated cell death has emerged as a promising therapeutic approach for treating cancer [3]. A previously undiscovered type of programmed cell death known as ferroptosis, which is distinctive from autophagy, necrosis, and apoptosis, was initially discovered in cancer cells with oncogenic Ras mutations [4]. Ferroptosis plays a role in the disorders of the neurological system, kidneys, and cardiovascular system and performs an integral function in cancers, including NSCLC [5–7]. Ferroptosis may be induced by a variety of agents, including drugs, chemical compounds, and small molecule drugs. Erastin, which is a cell-permeable piperazinyl-quinazolinone substance, is one of the compounds that is utilized extensively in the investigation of the molecular processes behind ferroptosis [8]. Erastin can produce iron accumulation and lipid peroxidation by interfering with several sites, such as the glutathione peroxidase 4 (GPX4) and the cystine/glutamate exchange transporter (SLC7A11).

Even though it has only been recently discovered that various regulators are responsible for modulating erastin-mediated ferroptosis in a variety of experimental settings, the key modulator of lipid metabolism in ferroptosis of cancerous cells is still not well comprehended. In 2002, a mutation in a gene called acyl-CoA synthetase long-chain family member 4 (ACSL4) was found to be the cause of the non-specific X-linked mental retardation [9]. ACSL4 had a substrate predilection for arachidonic acid (AA) and eicosapentaenoic acid (EPA). Even more intriguing is the fact that the levels of free AA may, in turn, influence the levels of ACSL4 protein within the cells [10]. To this day, it has been shown that ACSL4 dysregulation is linked to many illnesses, which include diabetes, acute kidney injury, and malignant tumors [7, 11, 12]. Recent research has shown that ferroptosis and the dysregulation of ACSL4 are strongly connected [13]. ACSL4 knockdown was shown to suppress erastin-mediated ferroptosis in HL-60 and HepG2 cells, whereas the upmodulation of ACSL4 was found to reestablish the susceptibility of K562 and LNCaP cells to erastin [9]. As a consequence, the levels of ACSL4 expression could be linked to the progression of NSCLC because of its role in triggering ferroptosis. Nonetheless, neither the expression profiles nor the roles of ACSL4 in NSCLC have been investigated to this point. Hence, the present research sought to examine the ACSL4 expression in NSCLC and its link to the clinical-pathological characteristics and patients' prognoses, as well as the involvement of ACSL4 in ferroptosis through experimental and bioinformatic analyses.

RETRACTED

## 2. Material and Methods

### 2.1. Bioinformatics Analyses of ACSL4

To begin, the Oncomine database (https://www.oncomine.org/) was retrieved in order to make a prediction about the level of ACSL4 mRNA expression found in lung cancer samples and normal samples. Next, the Cancer Genome Atlas (TCGA) LUAD and LUSC database was retrieved to evaluate the link between ACSL4 mRNA expression and clinical prognostic outcomes of NSCLC patients based on the data from UALCAN (http://ualcan.path.uab.edu/). In The Human Protein Atlas (HPA) (https://www.proteinatlas.org), the immunohistochemical (IHC) image was utilized to perform a comparative evaluation of the levels of ACSL4 protein expression between human NSCLC samples and normal samples. The prognostic utility of ACSL4 mRNA expression was investigated with the use of an electronic database referred to as Kaplan-Meier (KM) plotter (https://kmplot.com/analysis/). cBioPortal (http://www.cbioportal.org/) was employed to conduct an analysis of ACSL4 coexpression genes based on the TCGA-LUAD and LUSC datasets. To examine the ACSL4 functions, we utilized the GO and KEGG in the Database for Annotation, Visualization, and Integrated Discovery (DAVID) (https://david.ncifcrf.gov/).

### 2.2. Human Lung Cancer Samples

From 2018 to 2019, we recruited 36 NSCLC patients (18 cases of ADC and 18 cases of SCC) at the Sun Yat-sen University Cancer Center. For the subsequent real-time PCR tests, samples of tumor tissues and surrounding tissues that were five centimeters distant from the margin of the cancerous tissues were collected. Before receiving surgery, these participants did not undergo any adjuvant treatment, like radiotherapy, chemotherapy, or any other kinds of treatment. This research was subjected to approval by the Academic Committee of the Cancer Center at Sun Yat-sen University Cancer Center, and each patient gave their informed consent before taking part in the research.

### 2.3. Cell Culture and Treatment

The human lung cancer cells A549 and SPC-A-1 cell lines were procured from the American Type Culture Collection (ATCC; Manassas, VA, USA). Next, we cultured the A549 cells in Gibco™ Dulbecco's modified Eagle's medium (DMEM; Thermo Fisher Scientific, Inc., Paisley, UK), whereas the SPC-A-1 cells were grown in Roswell Park Memorial Institute 1640 Media (RPMI 1640; Gibco, USA) comprising 10% fetal bovine serum (FBS), 100 U/ml of penicillin, and 0.1 mg/ml of streptomycin (Thermo Fisher Scientific, Inc.) in a humid incubator with 5% CO_2_ and 37°C culture environment. A549 cells were subjected to treatment with 5 *μ*M erastin (Sigma-Aldrich, St. Louis, MO, USA) for 24 hours for the purpose of performing subsequent relevant analyses. Following that, the cells were collected in the manner detailed below in preparation for further examination.

RETRACTED

### 2.4. Cell Proliferation

An evaluation of the capacity for cells to proliferate was carried out with the aid of a Cell Counting Kit-8 assay (CCK-8, Sigma-Aldrich; Merck KGaA, Darmstadt, Germany) in compliance with the specifications stipulated by the manufacturer.

### 2.5. Quantitative Real-Time PCR Analysis

Synthesis of first-strand cDNA was accomplished following the guidelines provided by the manufacturer of the Reverse Transcription System Kit (OriGene Technologies). cDNA obtained from the cells was amplified utilizing the appropriate primers (ACSL4: 5′-GCTATCTCCTCAGACACACCGA-3′ and 5′-AGGTGCTCCAACTCTGCCAGTA-3′), and the data were normalized to actin RNA (5′-CACCATTGGCAATGAGCGGTTC-3′ and 5′-AGGTCTTTGCGGATGTCCACGT-3′).

### 2.6. RNA Interference and Gene Transfection

OriGene Technologies supplied the human ACSL4-cDNA used in this study. The Lentivirus Transduction System (Sigma) or the Lipofectamine™ 3000 (Invitrogen) was used to carry out the transfections following the guidelines provided by the respective manufacturer.

### 2.7. Iron Assay

In order to conduct the iron assay, we made use of an Iron Assay Kit (Sigma Aldrich, Milwaukee, WI, USA) to assess the level of total iron present per cell line. Subsequently, in a short time, 2 × 10^6^ cells were quickly homogenized in a range of 4 to 10 volumes of iron assay buffer. The insoluble material was separated from the samples by centrifuging them at a rate of 13,000 × g for 10 minutes at a temperature of 4°C. Iron reducer (in a volume of 5 *μ*l) was introduced into each sample well so that Fe^3+^ could be converted to Fe^2+^ to measure total iron. After the samples were well agitated by pipetting or with a horizontal shaker, the solutions were subjected to incubation for 30 minutes in the darkness at ambient temperature. Thereafter, 100 *μ*l of iron probe were introduced into each well that contained either a standard sample or a test sample. Once the samples were well agitated either by pipetting or with a horizontal shaker, the solutions were allowed to incubate for 60 minutes at ambient temperature in the darkness. At last, the absorbance was evaluated at 593 nm.

RETRACTED

### 2.8. Lipid ROS Assays

In order to analyze lipid ROS, the cells were first trypsinized before resuspension in a medium supplemented with 10% FBS. After that, 10 *μ*M of C11-BODIPY (Thermo Fisher Scientific, Inc.) was introduced into the samples before incubating them for 30 minutes at 37°C with 5% CO_2_, in the darkness. To get rid of any residual C11-BODIPY, the cells were rinsed two times in PBS. By employing a flow cytometer (Beckman Coulter Inc., Brea, CA, USA), the fluorescence of C11-BODIPY 581/591 was quantified by simultaneously recording red signals and green signals.

### 2.9. Statistical Analysis

GraphPad Prism 6.0 (GraphPad Software, Inc., USA) and SPSS 22.0 (IBM SPSS, Chicago, IL) were utilized to conduct all analyses of statistical data in this study. The results obtained from statistical analyses are presented as means ± SD. We examined whether there were significant differences across the groups with the help of the two-tailed Student's *t*-test or one-way analysis of variance (ANOVA) test. The threshold for significance was set at a *p* value < 0.05.

## 3. Results

### 3.1. ACSL4 Expression Is Downmodulated in Lung Cancer

We began by retrieving the Oncomine database, where we discovered that the level of ACSL4 mRNA expression in lung tumor samples was considerably lowered in contrast with that in normal samples (Figure 1). A tissue qPCR was undertaken to determine the expression of ACSL4 in postoperative lung tumor samples relative to normal lung samples. The findings illustrated that the relative ACSL4 expression level was remarkably lowered in tumor samples (*n* = 18) in contrast with the normal samples (*n* = 18) (*p* < 0.001, Figures 2(a) and 2(b)). After that, we scrutinized the HPA dataset to ascertain ACSL4 protein expression. It was discovered that normal lung tissues showed intense staining for ACSL4 (Figure 2(c)). Conversely, it was demonstrated that all malignant tissues had weak staining for ACSL4 (100%, 12 of 12 cases). In addition, the staining was predominantly present in the cytoplasm and the cell membrane (Figures 2(d) and 2(e)). The findings matched up perfectly with those found in the TCGA database (Figure 3(a)).

### 3.2. Decreased ACSL4 mRNA Expression Is Associated with Malignant Clinical-Pathological Characteristics in NSCLC Patients

In the current investigation, we examined whether there was a correlation between the expression of ACSL4 mRNA and clinical and pathological characteristics. In both ADC and SCC patients, the findings illustrated that ACSL4 mRNA expression was linked to the cancer stages, smoking behaviors, and the status of nodal metastases (*p* < 0.001, Figure 3). KM curves of overall survival (OS) and relapse-free survival (RFS) were constructed premised on the survival data obtained from the KM plotter to investigate the link between ACSL4 mRNA expression and NSCLC patients' prognoses. According to the findings, patients with ADC who had a high level of ACSL4 expression experienced considerably better OS and RFS (*p* = 0.007, *p* = 0.026, correspondingly, Figures 4(a) and 4(b)). Additionally, patients with SCC who had a high level of ACSL4 expression experienced exhibited an improved OS and RFS, whereas the differences did not meet the significance threshold (*p* = 0.16, *p* = 0.13, correspondingly, Figures 4(c) and 4(d)).

RETRACTED

### 3.3. Overexpression of ACSL4 Promotes Ferroptosis

We transfected ACSL4 cDNA into SPC-A-1 and A549 cells to ascertain the potential of ACSL4 expression to modulate the anticancer function of erastin (inducer of ferroptosis) in lung cancer (Figure 5(a)). Gene transfection was used to overexpress ACSL4, which resulted in a considerable enhancement of the susceptibility of SPC-A-1 and A549 cells to the erastin-mediated cell death (Figures 5(b) and 5(c)), indicating that ACSL4 is a necessary part of the ferroptosis-related regulatory mechanism. Both the peroxidation of lipids and the accumulation of iron are necessary elements in the process of ferroptosis activation. As a result, we examined whether ACSL4 affected these events during ferroptosis. Erastin caused a considerable increase in the generation of lipid ROS when ACSL4 was upregulated (Figure 5(d)). On the other hand, the upmodulation of ACSL4 did not have any effect on the erastin-mediated accumulation of iron (Figure 5(e)). Based on these data, ACSL4 may be a factor contributing to erastin-mediated ferroptosis through modulating lipid peroxidation; however, it does not seem to be a contributor to iron accumulation.

### 3.4. GO Functional Annotation and Pathway Enrichment of ACSL4

To investigate the fundamental process of ACSL4's participation in the pathologically aggressive biological behavior of lung cancer, we conducted a TCGA-LUAD and LUSC gene coexpression network analysis. We identified the remarkably coexpressed genes with ACSL4 in TCGA-LUAD and LUSC by utilizing the cBioPortal of Cancer Genomics. A criterion of absolute Spearman's *r* of ≥0.5 was utilized to determine whether genes in LUAD and LUSC were coexpressed with ACSL4, and the findings illustrated a coexpression of ACL4 with 56 genes in LUAD and 63 genes in LUSC. After that, these genes were entered into DAVID so that additional GO analysis and KEGG pathway analysis could be undertaken.  Table 1 contains a list of the three most significant terms derived from the GO functional annotation and the KEGG pathway enrichment analysis. The ubiquitin-induced proteolysis pathway was the one that was most relevant for the gene enrichment that occurred as a result of ACSL4 coexpression. Protein ubiquitination (GO: 0016567) and ubiquitin-protein transferase activity (GO: 0004842) accounted for the substantial proportion of enriched GO categories in the biological process and molecular function. In the cellular component ontology, the endocytic vesicle (GO: 0030139) ranked at the top in the pathophysiological process.

RETRACTED

## 4. Discussion

Ferroptosis was not discovered until 2012 when Dixon et al. published their findings on a study they had conducted on a small compound known as erastin [4]. The process of ferroptosis is a novel kind of regulated cell death that is reliant on iron and is linked to oxidative stress [14]. The typical characteristics of ferroptosis encompass lipidic and cytoplasmic accumulation of ROS, a decrease in the volume of mitochondria, an enhancement in the density of the mitochondrial membrane, rupture or loss of mitochondrial cristae, and rupture of the mitochondrial outer membrane [4, 15]. Following gene scanning using genome-wide CRISPR and microarray analyses of anti-ferroptosis cell lines, it was recently shown that ACSL4 is a significant factor involved in the ferroptosis process [13]. In the current investigation, the patterns of ACSL4 expression, as well as the clinical and pathological characteristics of NSCLC patients, were analyzed. Furthermore, we present the substantiation that ACSL4 is implicated in the accumulation of lipid intermediates in the process of ferroptosis. The degree of cellular susceptibility to the ferroptosis caused by erastin is correlated with ACSL4 expression. Mechanistically, it is conceivable that the ubiquitin-mediated proteolysis pathway is necessary for the ferroptosis that is triggered by ACSL4.

According to several reports, ferroptosis has a very strong correlation with a variety of human disorders [15, 16]. However, there has not been much research done on ferroptosis in NSCLC. Lai and his colleagues found that ferroptosis as an antitumor factor is inhibited in NSCLC [17]. In Li's study, NSCLC cells possessing chemotherapy based on cisplatin-resistant characteristics (N5CP cells) were acquired from the surgical excision of clinical samples taken from patients suffering from NSCLC [18]. They discovered that stimulation of the Nrf2/SLC7A11 pathway was closely linked to the resistance of cells to the cisplatin-based chemotherapeutic treatment. As a consequence, the modulation of Nrf2 or SLC7A11 expression by erastin or sorafenib can make tumor cells more or less sensitive to the treatment that is on the basis of cisplatin. Both erastin and sorafenib, which are both small compounds, successfully triggered ferroptosis in N5CP cells. This process was facilitated by the accumulation of lipid ROS within the cells. In addition, to successfully induce N5CP cell ferroptosis, modest dosages of erastin or sorafenib might be employed in conjunction with chemotherapeutic treatment premised on cisplatin. Accordingly, ferroptosis inducers such as sorafenib and erastin might be deemed as a new therapeutic regimen for patients who have NSCLC, especially individuals whose chemotherapeutic regimen was unsuccessful due to the use of cisplatin [18].

RETRACTED

Through its role as a central marker and modulator of ferroptosis, ACSL4 also performs an indispensable function as a crucial factor of ferroptosis susceptibility by modifying the lipid content of the cells [7]. ACSL4 deletion cells exhibited resistance to lipid peroxidation as well as ferroptosis [9]. Ferroptosis was partially caused by the formation of 5-hydroxyeicosatetraenoic acid (5-HETE), which was mediated by ACSL4. The generation of 5-HETE was attenuated by zileuton's pharmacological suppression, which inhibited ACSL4 upregulation-mediated ferroptosis [10]. ACSL4 increases the level of long polyunsaturated *ω*6 fatty acids that are present in cell membranes. In addition, ACSL4 is selectively expressed in a group of breast cancer cell lines that have a basal-like phenotype, which is predictive of the cell lines' susceptibility to ferroptosis [19]. Deletion of ACSL4 in prostate cancer (PCa) cells that express endogenous ACSL4 results in the attenuation of cell capacity to proliferate, migrate, and invade, whereas ectopic production of ACSL4 in ACSL4-negative PCa cells results in an enhancement of the proliferative, migratory, and invasive capacity of cells [20]. According to the findings of the research, ACSL4 is responsible for the upmodulation of many different pathway proteins, including *β*-catenin, LSD1, and p-AKT [20]. As a consequence of this, ACSL4 is considered to be a sensitive modulator of the ferroptosis process. On the other hand, ACSL4 has not yet been explored in ferroptosis-linked NSCLC. In this research, we discovered that the expression of ACSL4 was reduced in tumors and that this reduction was associated with an unfavorable prognosis. These findings imply that ACSL4 might function as a biological marker and a possible treatment target for NSCLC.

RETRACTED

Ferroptosis, like other types of cell death, is intimately linked to particular signaling pathways. The incidence of ferroptosis is tied closely to the accumulation of iron and the oxidation of lipids, which are the two most important components in the process [14]. To determine whether or not ACSL4 has a function in ferroptosis in NSCLC, an ACSL4 upregulation plasmid was introduced into two distinct NSCLC cell lines and subjected to transfection. According to the findings, ACSL4 overexpression may aggravate erastin-mediated cell death and increase the formation of lipid ROS. Conversely, the expression of ACSL4 did not affect the iron accumulation that was caused by erastin. As a fatty acid activating enzyme, the preferred substrates of ACSL4 are long-chain polyunsaturated fatty acids, including EPA and AA. ACSL4 is responsible for the catalysis of these fatty acids and the synthesis of the associated coenzyme A [10], both of which affect the process of lipid peroxidation.

Besides exploring the interaction that occurs between ferroptosis and other different kinds of cell death, it is also necessary to research the role and assess the molecular and pathway components that are connected to ferroptosis. Various recently discovered proteins, including metallothionein-1G, NCOA4, and PEBP1, have been linked to ferroptosis via the processes of the metabolism of iron and the peroxidation of lipids [21–23]. GO and KEGG analyses found that the gene coexpressed with ACSL4 is enriched in the pathway of protein ubiquitination. BAP1 is responsible for encoding a nuclear deubiquitinating enzyme that helps minimize ubiquitination of histone 2A on chromatin. Recent research has shown that the protein BAP1 reduces H2Aub occupancy on the regulator of the ferroptosis inhibitor SLC7A11 and suppresses the expression of SLC7A11 in a deubiquitinating-dependent way and that increased lipid peroxidation and ferroptosis are the direct results of BAP1's suppression of SLC7A11 expression, which impairs cystine absorption [24]. Moreover, BAP1 partially prevents the progression of tumors via SLC7A11 as well as ferroptosis, and cancer-related BAP1 mutants end up losing their capacities to suppress SLC7A11 and to stimulate ferroptosis [25]. The findings of this research indicate that, in addition to SLC7A11 ubiquitination, ACSL4 ubiquitination might well be implicated in the ferroptosis process, which warrants further investigation.

Additional research on ferroptosis is considered necessary not only to shed light on the mechanistic explanation behind the process but also to open the door to the possibility of developing novel therapeutic approaches. Sorafenib resistance, for instance, has been demonstrated to be the outcome of the metallothionein-1G-mediated suppression of ferroptosis during therapy for metastatic hepatocellular carcinoma [21]. In a group of human cell lines derived from a variety of cancerous tissues, Lachaier et al. examined the levels of ferroptosis that were caused by sorafenib and compared them to the levels that were induced by the standard compound, erastin [26]. They discovered that sorafenib promoted ferroptosis in kidney carcinoma cell lines. In addition to this, they discovered that the ferroptotic potency of sorafenib was positively correlated with that of erastin. Sorafenib is the only medication that can achieve ferroptotic efficacy in comparison to other kinase inhibitors, which makes sorafenib the first anticancer treatment to be licensed for use in the clinical setting that can trigger ferroptosis [26]. Doll et al. additionally illustrated that pharmacologically targeting ACSL4 using the antidiabetic compound class, thiazolidinediones, and alleviates tissue death in mice ferroptotic model, implying that inhibiting ACSL4 might be a useful therapeutic strategy for the prevention of illnesses linked to ferroptosis [13].

RETRACTED

## 5. Conclusion

Our research illustrated that the expression level of ACSL4 is lowered in NSCLC, which was shown to have a correlation with the clinical and pathological characteristics of patients. By stimulating ferroptosis, ACSL4 can partially inhibit the growth of NSCLC cells. These findings suggest that ACSL4 might be considered a viable treatment target for NSCLC, providing a foundation for future research on clinical pathways that involve ACSL4.

## Figures and Tables

**Figure 1:** The Oncomine database indicates that NSCLC tissues had low levels of ACSL4 mRNA expression. An investigation of ACSL4 mRNA levels was carried out by retrieving the Oncomine database for (a) overall cancer type, (b–d) ADC, and (e–g) SCC grouped by NSCLC and normal lung tissue. All *p* < 0.001 vs. control.

**Figure 2:** Compared with normal lung samples, NSCLC tissue samples showed a considerable reduction in ACSL4 expression. (a, b) A qPCR was utilized to examine ACSL4 mRNA expression in 18 pairs of NSCLC and corresponding neighboring normal lung tissues. ACSL4 IHC demonstrated strong staining in normal lung tissues (c); weak staining in NSCLC tissue (d, e). ^∗∗∗^*p* < 0.001 vs. control.

**Figure 3:** Levels of ACSL4 mRNA expression in patients suffering from NSCLC that were included in the TCGA dataset cohorts. (a, e) A comparison of the ACSL4 expression in ADC and SCC tissues with that of normal controls is depicted in the plot chart. (b–d) Plots chart illustrating the expression of ACSL4 mRNA between cancer stages, smoking habits, and nodal metastasis status in ADC patients. (f–h) Plots chart illustrating the expression of ACSL4 mRNA between cancer stages, smoking habits, and nodal metastasis status in SCC patients. ^∗∗∗^*p* < 0.001 vs. control.

RETRACTED

**Figure 4:** Patients diagnosed with NSCLC who had high levels of ACSL4 expression attained a better chance of survival. (a, b) Overall survival (OS) and recurrence-free survival (RFS) were analyzed utilizing Kaplan–Meier curves for all patients diagnosed with ADC. (c, d) Kaplan–Meier curves of OS and RFS for all cases of SCC.

**Figure 5:** Upmodulation of ACSL4 enhances ferroptosis. (a) mRNA expression of ACSL4 after transfection in specified cells. (b, c) In A549 and SPC-A-1 cells, upregulation of ACSL4 enhanced erastin-induced cell death. (*n* = 3, ^∗∗∗^*p* < 0.001 vs. control cDNA group). (d, e) After 24-hour treatment with erastin, lipid ROS and iron in A549 and SPC-A-1 cells were measured (*n* = 3, ^∗∗^*p* < 0.01 vs. control cDNA subgroup).

**Table 1:** Gene Ontology and pathway enrichment analysis of the ACSL4 coexpressed genes in TCGA-LUAD and LUSC.

Ontology	ID	Description	*p* value	*p*.adjust	*Q* value
BP	GO:0016567	Protein ubiquitination	1.52*e*-04	0.040	0.031
BP	GO:0032446	Protein modification by small protein conjugation	1.57*e*-04	0.040	0.031
BP	GO:0007265	Ras protein signal transduction	1.76*e*-04	0.040	0.031
CC	GO:0030139	Endocytic vesicle	1.10*e*-04	0.015	0.012
CC	GO:0044322	Endoplasmic reticulum quality control compartment	1.28*e*-04	0.025	0.015
CC	Go:0031461	Cullin-RING ubiquitin ligase complex	1.42*e*-04	0.025	0.015
MF	GO:0004842	Ubiquitin-protein transferase activity	2.30*e*-05	0.002	0.001
MF	GO:0005095	GTPase inhibitor activity	1.74*e*-04	0.025	0.015
MF	GO:0019003	GDP binding	2.63*e*-04	0.032	0.022
KEGG	03050	Ubiquitin-mediated proteolysis	1.13*e*-05	5.43*e*-04	2.38*e*-04
KEGG	04141	Protein processing in endoplasmic reticulum	8.53*e*-04	0.008	0.003
KEGG	04114	Oocyte meiosis	9.00*e*-04	0.008	0.003

## Data Availability

The simulation experiment data used to support the findings of this study are available from the corresponding author upon request.
